# Percutaneous Intervention of Iatrogenic Iliac Artery Vascular Complication

**DOI:** 10.7759/cureus.10181

**Published:** 2020-09-01

**Authors:** Sabah Siddiqui, Sergey Ayzenberg, Ahmad Morshed, Avraham Miller, Yury Malyshev

**Affiliations:** 1 Cardiology, Maimonides Medical Center, Brooklyn, USA

**Keywords:** percutaneous endovascular repair, retroperitoneal hemorrhage, lmca, complex pci, covered stents

## Abstract

The mortality of patients from a retroperitoneal hematoma remains high if treatment is delayed or inappropriate. Percutaneous endovascular repair of iatrogenic vascular complications is quickly becoming the treatment of choice. Here, we report a case of a 76-year-old female with a non-ST-elevation myocardial infarction, whose cardiac catheterization revealed a 70% distal left main coronary artery (LMCA) stenosis. She underwent successful rotational atherectomy and deployment of drug-eluting stents of the distal LMCA. Following percutaneous coronary intervention, she suffered acute profound hypotension and was found to have a retroperitoneal hematoma. Given the high cardiac risk for vascular surgery due to recent intervention and overall comorbidities, she was immediately taken to the cardiac catheterization laboratory and had a diagnostic angiogram, which revealed a right external iliac artery perforation that was treated with a covered stent. She tolerated the procedure well. This case highlights the importance of early diagnosis of retroperitoneal bleed, the prompt decision to take the patient to the cardiac catheterization laboratory, and potential use of intravascular interventions to ensure a successful outcome.

## Introduction

Cardiac catheterization and percutaneous intervention can result in vascular access-site complications. A retroperitoneal hemorrhage is a potential life-threatening complication of femoral artery puncture that should be suspected in any post-catheterization patient who develops hypotension, ipsilateral flank, abdominal or back pain, or a drop in hemoglobin without a source [1]. Hemodynamically stable patients can usually be managed with fluid resuscitation, blood transfusion, or a correction of coagulopathy [2]. Percutaneous endovascular repair of vascular complications (VCs) is quickly becoming the treatment of choice for various reasons, which are outlined below. Surgical open repair of retroperitoneal bleeding vessels can be reserved for cases when there is failure of conservative or endovascular measures to control the bleeding. In addition, surgical repair may also be required if endovascular facilities or expertise is unavailable. The mortality of patients with retroperitoneal hematoma remains high if treatment is delayed or inappropriate [2]. Therefore, it is of utmost importance that VC post-interventional procedures be recognized in a timely fashion and the prompt treatment could benefit in improved mortality. There are only a few cases in the literature describing the use of covered stents (CS) to manage a retroperitoneal bleed in the cardiac catheterization laboratory (CCL) post-complex high-risk percutaneous coronary intervention (PCI).

## Case presentation

A 76-year-old female with known coronary artery disease and chronic kidney disease stage IV (baseline estimated glomerular filtration rate of 22) was admitted to our facility with episodes of intermittent, exertional, chest pain for two weeks. Her electrocardiogram (ECG) showed normal sinus rhythm with poor R wave progression and her plasma troponin levels increased from 0.01 to 0.19 ng/mL (normal value is < 0.04 ng/mL). She was treated for non-ST-elevation myocardial infarction and underwent left heart catheterization. This revealed a distal left main coronary artery (LMCA) stenosis of 70%, and a left anterior descending artery (LAD) with 85% heavily calcified proximal and 90% mid disease (Figure 1).

**Figure 1:** Diagnostic coronary angiography reveals a distal left main coronary artery (LMCA) stenosis of 70% (red arrow), a left anterior descending artery (blue arrow) with 85% heavily calcified proximal and 90% mid disease, and 99% distal left circumflex (yellow arrow) disease

The left circumflex artery (LCx) had a 99% distal stenosis. The right coronary artery (RCA) had a proximal 40% lesion. After an extensive discussion, given her age and other comorbidities she was deemed to be a poor surgical candidate. The decision was made to proceed with PCI of the LMCA and LAD with preparation of the lesion with the Rotablator™ (Boston Scientific, Marlborough, MA) rotational atherectomy system. 

The right femoral artery was accessed using an ultrasound assist and 7 French (Fr) sheath was inserted. The patient has an opening aortic pressure of 161/76 mmHg. She underwent successful rotational atherectomy of the distal left main artery into the proximal LAD with the deployment of Synergy Rx™ monorail 3.0 mm x 38 mm drug-eluting stent (Boston Scientific, Marlborough, MA). The patient also received a 2.5 mm x 28 mm Synergy Rx drug-eluting stent to the mid LAD (Figure 2).

**Figure 2:** Post-PCI LM stent into proximal LAD with TIMI 3 flow and excellent angiographic results PCI, percutaneous coronary intervention; LM, left main artery; LAD, left anterior descending artery; TIMI, thrombolysis in myocardial infarction

The proximal LAD and LCx were post-dilated with an Emerge™ Over-the-Wire (OTW) 3.0 mm x 12 mm balloon (Boston Scientific, Marlborough, MA). A preclosure femoral angiogram was performed, and the decision was made to deploy an 8 Fr Angio-Seal™ (St Jude Medical, St. Paul, MN) to the right femoral artery to achieve hemostasis. The patient had a closing aortic pressure of 163/81 mmHg and had remained hemodynamically stable throughout the procedure. Post-PCI, the patient was found to be transiently unresponsive, and when she regained consciousness, she was feeling weak and was slightly bradycardic. ECG did not reveal any changes, and an emergency transthoracic echocardiogram did not reveal any pericardial effusion and showed normal left ventricle (LV) and right ventricle (RV) systolic function. Her access site did not show an obvious hematoma. Urgent point of care labs showed a hemoglobin drop from 9.1 to 7.1 gm/dL (normal 12-16 gm/dL) and hypotension to a systolic blood pressure (SBP) of 54 mmHg, she was immediately transfused two units of packed red blood cells (PRBCs) and given protamine sulfate and there was an improvement in the SBP. In the meantime, she was taken for urgent CT scan that showed a moderate right-sided retroperitoneal hematoma along the plane of the right iliac artery (Figure 3).

**Figure 3:** CT image with moderate right-sided retroperitoneal hematoma (red arrow) along the plane of right iliac artery

Vascular surgery was also consulted. Given the high cardiac risk for vascular surgery due to recent high-risk PCI and overall comorbidities, the patient was taken emergently to CCL. Access was obtained via left femoral artery, a cross over sheath was placed, and a diagnostic angiogram revealed extravasation of contrast in the right external iliac artery (Figure 4).

**Figure 4:** Diagnostic angiography showing right external iliac artery perforation (red arrow)

Tamponade of the lesion was done with a Mustang 7.0 mm x 40 mm OTW balloon (Boston Scientific, Marlborough, MA), which was subsequently covered with a 6 mm x 5 cm Viabahn® covered stent (WL Gore and Associates, Newark, DE) with confirmation of no further extravasation of contrast (Figure 5).

**Figure 5:** Post-balloon tamponade and placement of covered stent in the right external iliac artery into the common femoral artery

A CT scan performed two days later showed an interval mild decrease in size in right-sided retroperitoneal hematoma and right pelvic sidewall right groin hematoma. In addition, the patient did not require any more units of PRBCs. Moreover, the patient was managed on an antiplatelet therapy of aspirin 81 mg once a day and clopidogrel 75 mg once a day which she tolerated well. There was a transient worsening in the chronic kidney disease with the return of renal function to baseline at discharge 10 days later.

## Discussion

Percutaneous endovascular repair of VCs is quickly becoming the preferred therapeutic intervention, especially for patients who cannot tolerate vascular surgery due to advanced cardiovascular disease (CVD) [3]. Aortic bifemoral bypass is an established method of treatment of peripheral vascular disease such as iliac artery disease depending on the type of lesion [4,5]. Surgical cutdown and suture of the access site is a treatment for aortic pathologies, such as traumatic injury [6]. However, surgical treatment is burdened with a higher proportion of perioperative complications (5% to 10% of early complications) and higher mortality than endovascular treatment. When compared to surgery, endovascular treatment is less invasive, with easy percutaneous access to iliac arteries and a faster bleeding exclusion [7]. Immediate endovascular treatment in the catheterization lab ensures lower complication rate, and bypasses transportation to the operating room and general anesthesia, thus saving crucial time, particularly in retroperitoneal bleeding cases. It also reduces the overall length of hospital stay. More importantly, this technique reduces exposure to the risks of general anesthesia in a group of patients who are often affected by advanced CVD [3]. In the above presented case, our patient had just undergone a complex high-risk PCI and given her age and overall comorbidities, the patient was deemed a high cardiac risk for surgery. Once the retroperitoneal bleed was identified, the quick decision to take the patient immediately to the CCL for a prompt diagnosis to localize the perforation site and subsequent intervention was helpful in achieving a positive outcome.

The various percutaneous options to treat VCs include the use of prolonged balloon tamponade, CS or stent grafts, coil embolization, vascular plug, coagulated thrombus injection, and localized thrombin injection of pseudoaneurysms [8]. The endovascular repair of iatrogenic arterial injuries by means of CS has been proposed as a valuable alternative to surgical repair. CS combines a self-expanding stent with expanded polytetrafluoroethylene and aims to reduce in-stent restenosis and distal embolization by preventing the ingrowth of neointimal tissue into the stent and covering the ulcerated segments of vessels. Contoured proximal edge, heparin bioactive surface, and the introduction of 5-mm-diameter stent graft all aim to reduce the risk of edge stenosis and stent thrombosis [9]. 

However, for a few cases [10,11], there is not much reported in the literature regarding percutaneous management of iatrogenic iliac artery perforations. Once such case series reported 13 patients with iatrogenic arterial iliac ruptures that were treated with stent grafts [7]. Another case showed successful treatment of a large iliac artery rupture with a coated stent [12]. Arat and colleagues [13] reported successful treatment of a femoral bleeding site with two covered self-expanding coronary stent grafts. These were shown to be done in a minimally invasive, efficient, and safe method and had satisfactory short- and mid-term results [14]. CS for the treatment of traumatic arterial injuries offer a promising alternative to conventional operative repair with comparable patency and less major morbidity and mortality [15].

Percutaneous transluminal angioplasty with CS may be complicated by abrupt occlusion, deformation, and kinking, and loss of vessel branches after stenting and restenosis [16]. This may be minimized by appropriate patient selection, minimizing collateral coverage, and anti-thrombotic medications. It remains unclear if the potential advantages of CS outweigh the risks for patients with long segment disease, where it competes primarily with open bypass surgery [2]. Therefore, further studies with larger populations are needed to confirm these preliminary findings and to evaluate the long-term durability of CS in such circumstances [16].

## Conclusions

Percutaneous treatment for iatrogenic VCs such as retroperitoneal bleeding allows for reduced morbidity. It is a rapid, less invasive form of management with the possibility to treat patients with multiple comorbidities, which is essential in achieving overall improvement in mortality. With the above case, we have demonstrated the successful use of balloon tamponade followed by placement of a CS to seal an iatrogenic endovascular iliac artery perforation in a patient who had just undergone a complex high-risk PCI. Given advanced CVD, age and overall comorbidities the patient was high cardiac risk for surgery. Therefore, once the retroperitoneal bleed was identified, the prompt decision to take the patient to the catheterization lab to diagnose and intervene on the perforation was essential in saving invaluable time and ensuring a successful outcome. 
